# The Effect of a New Ligation and Venipuncture Method on Vena Basilica Vessel

**DOI:** 10.1155/2022/9384983

**Published:** 2022-05-14

**Authors:** Yuanhong Mao, Xiaomei Huang, Hong Yang, Shu Zhou, Aihong Yuan, Gang Lin, Guiling Geng

**Affiliations:** ^1^Medical Imaging Department, Nantong First People's Hospital, Jiangsu, China; ^2^Radiotherapy Department, Nantong First People's Hospital, Jiangsu, China; ^3^Internal Medicine-Cardiovascular Department, Nantong First People's Hospital, Jiangsu, China; ^4^School of Nursing, Nantong University Medical School, Jiangsu, China

## Abstract

**Objective:**

This study evaluated the impact of a novel venipuncture method on vascular parameters of vena basilica to provide a new technical option for the clinical management of difficult venipuncture.

**Methods:**

32 volunteers examined by ultrasound at the Medical Imaging Center of The First People's Hospital of Nantong, Jiangsu province, from February 2020 to April 2020 were randomly selected. One hand of each patient was ligated with the traditional single tourniquet and the new ligation method for 20 seconds. Then, the distance between the left or right vena basilica and the skin and the diameter of blood vessels were measured by ultrasound. 98 patients with peripheral venipuncture difficulty who were examined by ultrasound of a third-grade hospital from April 2019 to March 2020 were selected and randomly divided into control group (*n* = 49) and experimental group (*n* = 49). The traditional method was used in the control group, and the new peripheral venipuncture was used in the experimental group. The success rate of single puncture, preparation time before puncture, time required for puncture operation, pain reaction during puncture, intravascular congestion after puncture, subcutaneous tissue injury, and vascular reuse rate after puncture were compared between the two methods.

**Results:**

The new ligation and puncture method increased the diameter of peripheral superficial vein vessels by 0.51 ± 0.04 mm, and the change of vena basilica diameter was not significantly associated with gender and age of patient. The success rate of single puncture and the vascular reuse rate were significantly higher in the experimental group than in the control group, while the preparation time and venipuncture time, as well as the patient's pain response, were significantly lower in the experimental group compared to the control group, and the intravascular congestion and subcutaneous tissue injury were lower. In addition, the mean satisfaction score of patients in the experimental group was higher than that of the control group.

**Conclusion:**

The new ligation and puncture method was an effective vena basilica dilation technique for filling the peripheral superficial veins, improving puncture success rate of peripheral difficult vein, and reducing patient pain, which was worth popularizing and applying in clinic.

## 1. Introduction

The establishment and use of vascular access was a widely used route of administration and treatment for outpatient, emergency, or inpatient patients [1]. According to the 2010 National Hospital Outpatient Survey in the United States, more than a quarter (35.2 million) of all emergency department visits in the United States require vascular access for parenteral administration [2]. The successful establishment of vascular access was the establishment of “life channel” for patients in critical condition, such as acute and critical patients, fasting, surgery, hemorrhagic shock, cardiac and respiratory arrest, and resuscitation. However, not all vascular access was successfully established on the first attempt.

However, venipuncture was one of the most challenging and common skills in diagnosis and treatment [3]. The lack of clearly visible and palpable veins was called difficult veins. In an evaluation of 147,260 patients, it was found that approximately 8.9% of patients had difficult venous access and associated delays in care, and the number of patients with difficult veins is increasing each year due to the increased prevalence of obesity, diabetes, etc. [4, 5]. Due to the progress of society, the increase in life expectancy, and the change of diet structure, there were more and more patients with obesity, diabetes, hypertension, and cancer after chemotherapy, and more and more patients with difficult veins. Therefore, establishing vascular access became a challenging operation [6]. For patients with difficult intravenous access (DIVA), puncture was difficult and took a long time. Difficult veins led to repeated attempts and multiple invasive punctures by nurses, which not only delayed diagnosis [7] and treatment but also increased the pain of patients, increased the negative emotions of patients and their families, and brought pain to patients [8]. Moreover, it led to the intensification of contradictions between nurses and patients, promoted the occurrence of violence, and affected the practice safety of medical staff [8, 9]. It caused pressure and challenges for nursing technicians involved in intravenous therapy [10], seriously damaged the physical and mental health of nursing staff, and caused demission, career change, and loss of nursing staff [11]. Whalen et al. [12] had shown that peripheral vascular access was one of the most common operations in the emergency department, and successful venipuncture was crucial for timely diagnosis and treatment. Difficulty in establishing vascular access was a real threat to patient safety.

In order to improve the one-time success rate of puncture veins, some scholars tried vein visualization technology (such as using the normal light, color Doppler ultrasound technique, near-infrared visualization techniques, vein imaging instrument [13–15]), and expansion techniques such as stimulation the impact surface vein [16] (gravity, clenched his fists, local extrusion and massage, and tourniquet technology); vasodilators such as nitroglycerin, gingerol, mucosaccharides sulfonate, and safflower oil were used locally [17, 18]. Other scholars did a lot of research and improvement on the puncture operation methods of difficult veins and improved the technique of venipuncture by ligation of double tourniquets [19]. However, there were some limitations to the above methods, such as increasing the operation time and steps, consuming manpower and material resources, and increasing expenses. Therefore, it was the most direct and effective solution to study a simple, easy, easy to master, easy to operate, and effective dilation of peripheral veins, which could effectively ensure timely intravenous administration and save patients' lives. The purpose of this study was to determine the effects of limb drooping at the venipuncture side, ligating double tourniquet, and loosening fist clenching on the depth and diameter of vena basilica and to verify the successful puncture effect of this method in patients with enhanced CT scanning difficult veins.

## 2. Materials and Methods

### 2.1. Patient Collection

Thirty-two volunteers, including 13 females and 19 males, underwent ultrasonography at the Medical Imaging Center of the First People's Hospital of Nantong city, Jiangsu Province, were selected. Inclusion criteria: (1) age ≥ 18; (2) able to answer questions correctly and complete instructions; (3) the patient can get a normal sitting position; (4) all subjects signed informed consent. Exclusion criteria: (1) patients with limitations due to trauma or change of body position; (2) patients with unstable vital signs; (3) patients with artificial airway mechanical ventilation; (4) patients with absence of upper limbs; (5) patients with coagulation and vascular wall diseases.

From April 2019 to March 2020, 98 patients with peripheral venipuncture difficulties underwent ultrasonography at the medical imaging center of a III grade hospital were selected. The patients were randomly divided into experimental group (*n* = 49) and control group (*n* = 49) depending on the method of venipuncture. Inclusion criteria: ① informed consent, age ≥ 18 years old, without coagulation and vascular wall diseases; ② the superficial veins were evaluated as grade III difficult veins according to the superficial vein vascular grading criteria of Chinese scholar Ning et al. [20]: (1) indistinct veins, hardened vessels, phlebitis, and inconspicuous superficial veins; (2) sliding fine veins; (3) collapsed veins (dehydration, shock, etc.); (4) other special parts of unclear small blood vessels; ③ clear mind, answer questions correctly, and cooperate to complete the command action; ④ the patient's condition permitted, could take the sitting or half decubitus position. Exclusion criteria: ① patients with good peripheral shallow filling and easy venipuncture success; ② there were skin infection, ulceration, hemiplegia, and limb side of the puncture site; ③ cervical vertebra or lumbar vertebra and other diseases should not be half decubitus; ④ patients with tracheotomy or endotracheal intubation and ventilator assisted ventilation; ⑤ all kinds of dementia or neurological diseases, unable to communicate with patients. The general information of patients is recorded. All patients signed an informed consent form, and this study was approved by the Nantong First People's Hospital Ethics Committee (2021KT108).

### 2.2. Ultrasound Examination

A traditional ligature single tourniquet and a ligature double tourniquet were applied to each subject for 20 seconds. The CHISON full digital color ultrasound system (Site-Rite∗80) was used to measure the vena basilica of patients. The distance of veins from the skin and the diameter of the blood vessels were measured.

Traditional ligation method: the subjects sat on the plastic steel chair for diagnosis and treatment, and their upper limbs were placed flat on the operating table, with soft pillows under their limbs. A tourniquet was tied to the proximal end 6 cm above the vessel to be measured. The tightness of the tourniquet was 3/4 of the circumference of the upper arm. The tourniquet was stretched and tied to the upper arm at a pressure of 4.0 kpa (30 mmHg). According to the stopwatch, 20 seconds later, measure the right or left vena basilica distance from the skin and blood vessel diameter. The measured limb was lifted for 2 minutes, and the above values were measured with the new ligation method after resting for 10 minutes.

New ligation method: the patient was seated in a plastic steel chair with the upper limb palm-facing up and the back of the hand resting on the ipsilateral knee. Make the patient take a comfortable posture of 45° prolapse of the puncture side limb. Apply the first tourniquet at the proximal end 6 cm above the measurement point. The tightness of the tourniquet was to stretch the tourniquet 3/4 of the circumference of the upper arm and tie it at a pressure of 4.0 kpa (30 mmHg) [10]. Apply the second tourniquet at the proximal end 8 cm above the puncture point with the same tightness as the first tourniquet (the distance between the two tourniquets is 2 cm). After the first tourniquet was tied, the patient was instructed to make a loose fist clench for 20 seconds (15/10 seconds). According to the stopwatch, 20 seconds later, measure the right or left vena basilica distance from the skin and blood vessel diameter.

### 2.3. Venipuncture Method

Control group: traditional peripheral venipuncture was used, and the patient was seated. On the puncture side, the upper limb was placed flat on the operating table, and the soft pillow was placed under the limb. A single tourniquet was applied 4-6 cm above the puncture point proximal to the heart (Figure 1(a)). The puncture site was either the elbow of the upper limb or the vein of the forearm. The closed venous indwelling needle (20 G × 1.16 IN, 1.1 mm × 30 mm, Suzhou Bidi Medical Instrument Co., Ltd.) was selected, and skin puncture with a sterile syringe and the steel needle was fixed, and the hose of the closed indwelling needle was sent along the vascular direction. Reconfirm that the indwelling needle was fixed intravascular with a 3 M transparent compress. The long catheter was washed with sterile 0.9% sodium chloride 3 ml pulse technique, and the sealing clip was clamped.

Experimental group: modified peripheral venipuncture was used. The patient was sitting in the diagnosis and treatment chair with the upper limb palm facing upwards and the back of the hand on the knee of the ipsilateral lower limb. Make the puncture on the side limb at 45° droop position. Using a new ligation method to tie the tourniquet (Figure 1(b)). The puncture position was the middle cubital vein, vena basilica, cephalic vein, and other thick peripheral veins. Insert a shallow venipuncture needle fin and take 10 to 20° to puncture the skin; slowly advance the needle toward a venous line direction. Fix the steel needle; the closed IV needle hose was slowly pushed in the direction of the vein. Reconfirm that the indwelling needle was fixed intravascular with a 3 M transparent compress. The long catheter was washed with sterile 0.9% sodium chloride 3 ml pulse technique, and the sealing clip was clamped (Figure 1(c)). Four senior N3 level nurses were trained and passed the examination, and the improved venipuncture method was used to perform peripheral vein puncture for patients with difficult veins.

### 2.4. Evaluation Indicators

The success rate of one-time puncture, preparation time before puncture, time required for puncture operation, pain reaction during puncture, intravascular congestion after puncture, subcutaneous tissue injury, and vascular reuse rate after puncture of the two groups were recorded and compared.

Success rate of one-time puncture: no repeated subcutaneous needles to detect blood vessels. Two or more punctures were recorded as successful catheterization after needle return or successful repuncturing after replacement of a new closed indwelling needle.

Time required for puncture operation: the time required for puncture operation referred to the period from selecting the vein to successfully fixing the catheter, rinsing the catheter, and clamping the catheter clamp.

### 2.5. Satisfaction

Questionnaires with the same contents were given to the experimental group and the control group at the end of venipuncture to investigate whether the patients were satisfied with the operation time and the operation effect. The satisfaction survey was conducted on a 10-point scale. A score of 10 meant very satisfied; 9, 8, and 7 were satisfied; 6 and 5 were fair; 4, 3, and 2 were not very satisfied; and 1 was very dissatisfied. After the intravenous indwelling needle puncture operation was completed, the patients chose their own score for satisfaction, and put the written score into the satisfaction box of the experimental group and the control group. After studying, the score was uniformly scored.

### 2.6. Statistical Treatment

SPSS 24.0 statistical software was used in this study. The measurement data conforming to normal distribution were represented by mean ± standard deviation (SD), and an independent sample *T* test was used. The measurement data that did not conform to normal distribution were represented by the median, and the difference between the two groups was compared by Mann–Whitney *U* test. Statistical data was expressed in percentage (%) or number (*n*), and *χ*^2^ test was used for analysis. *P* < 0.05 was considered statistically significant.

## 3. Results

### 3.1. Effect of Two Ligation Methods on Vessel Depth and Diameter

First, ultrasound was used to detect the effects of two ligation methods on vessel depth and diameter (Figures 2(a) and 2(b)). The results showed there was no statistically significant difference in blood vessel depth measured by the new ligation method compared with the conventional single tourniquet method. The blood vessel diameter measured by the new ligation method was significantly larger than the conventional single tourniquet method group (Table 1).

### 3.2. General Data of the Two Groups of Patients with Difficult Veins

A total of 49 patients (15 males and 34 females) in the control group were 64.00 ± 12.10 years old, while 49 patients (17 males and 32 females) in the experimental group were 62.49 ± 9.59 years old. There was no statistical difference between the two groups in age, gender, and the history of basic diseases (hypertension, diabetes, and tumor chemotherapy), indicating that the two groups were comparable (Table 2).

### 3.3. Comparison of Vessel Depth and Diameter in Patients with Difficult Veins

By using ultrasound, the effect of two ligation and puncture methods on vessel depth and diameter in patients with difficult veins was compared. The results revealed that, compared with the control group, the experimental group using the new ligation method had shallower depth of blood vessels and larger vessel diameter (Table 3). Such differences indicated that the new ligation method facilitated vascular puncture in patients with difficult veins.

### 3.4. Comparison of Related Evaluation Indicators between Two Ligations and Venipuncture Methods in Patients with Difficult Veins

The two different ligation and venipuncture methods were further evaluated. The success rate of one-time puncture in the experimental group was 95.9%, significantly higher than 73.5% in the control group. The time required for preparation before puncture and for puncture operation time was significantly reduced in the experimental group. During puncture, the experimental group was associated with less pain response. After puncture, significant improvement of intravascular congestion and subcutaneous tissue injury was found in the experimental group compared with the control group. In addition, the vascular reuse rate after puncture in the experimental group (85.71%) was significantly higher than that of the control group (63.27%) (Table 4). The above results indicated that the new ligation and venipuncture method could improve the venipuncture effect in patients with difficult vessels.

## 4. Discussion

With the acceleration of the aging process and high incidence of cancer, increasing patients require long-term parenteral nutrition, intravenous infusion, infusion of thick or high permeability liquid and chemotherapy drugs, and other patients. Such treatments are often based on venipuncture. However, in the elderly, the problem is more complicated by increases in vascular stiffness and fragility and slow venous return, which results in increased difficulty in puncture and even puncture failure [21]. Failure of puncture further leads to drug leakage, inducing phlebitis and even tissue necrosis [22]. Venipuncture also brings anxiety and pain to patients [23], enhancing the difficulty of clinical work and reducing the effect of treatment. Therefore, finding an effective and less painful venipuncture method is of vital significance.

Single tourniquet ligation is a traditional method for venipuncture, but it has unsatisfactory outcome in superficial venipuncture with poor vascular filling. Some scholars have used double tourniquet ligation and compared it with the traditional one and found that the former significantly improved venous filling and the success rate of venipuncture [24]. Some studies have shown that the optimal duration of tourniquet ligation for venipuncture is 40-120 s [12]. During venipuncture, ligating the tourniquet at the proximal end of the puncture site can increase the resistance of distal venous return, thus elevating the venous blood pressure and facilitating the filling of superficial veins. Ultrasound-guided indwelling needle puncture of peripheral veins contributes to the determination of vascular location in patients, increases in the scope of vein selections, and observation of the inner diameter of blood vessels and the depth from the body surface [25]. This study compared the depth and diameter of vessels in patients after single and double tourniquet ligation using ultrasound and found that vessel depth was shallow and vessel diameter increased in patients receiving the latter method, indicating vessel filling after double tourniquet ligation, which is consistent with exiting studies.

The new ligation and puncture method refers to arm dropping, double tourniquet ligation and loosening fist. Given the gravity, arm dropping has slower venous blood return than arm placing flat on a table after ligation, causing venous blood stasis in a short time and increasing the blood volume in the superficial vein distal to the tourniquet to fill the vessels. Loosening the fist can promote the filling of peripheral veins at the distal end of the tourniquet and enlarge vascular lumen, resulting in a significant sense of loss of air pressure resistance and rapid blood return [26]. The results of this study also showed that, compared with the traditional ligation and puncture method, the new one could significantly increase the success rate of one-time puncture in patients with difficult vessels, reduce vascular injury, and improve patient satisfaction. Previous studies adopted simple double tourniquet, simple limb drooping, or simple loosening fist to solve the problem of difficult venipuncture [21]. In this study, the three factors were combined together for the first time, and the synergistic and superimposed effects of the three factors played a positive role in the filling of peripheral superficial veins.

## 5. Conclusion

The new ligation and puncture method promoted the filling of peripheral superficial veins and increased the diameter of peripheral superficial veins, thus improving the puncture success rate of peripheral difficult veins and shortening the puncture operation time and relieving the pain of patients. It provides data support for improving the success rate of venipuncture clinically.

## Figures and Tables

**Figure 1:** Diagram of different ligation and puncture methods. (a) Traditional peripheral venipuncture; (b) operation diagram of the new peripheral venipuncture; method (c) operation diagram of the new puncture method for difficult vein.

**Figure 2:** Ultrasound detection on the effect of two ligation methods on vessel depth and diameter. (a) Images of vascular depth and diameter measured by conventional methods; (b) images of vessel depth and diameter measured by the new ligation method.

**Table 1:** Comparison of vessel depth and vessel diameter between two tourniquet fastening methods.

Parameter	Conventional single tourniquet method	New ligation method	*z*/*t*	*P*
Blood vessel depth	5.00 (3.42, 6.55)	4.01 (3.21, 7.97)	1.765	0.078
Blood vessel diameter	4.54 ± 1.05	5.05 ± 1.09	4.347	0.001

Data was expressed as mean ± SD or median.

**Table 2:** General data of the two groups of patients with difficult veins.

Projects	Control group (*n* = 49)	Experimental group (*n* = 49)	*t*/*χ*^2^	*P*
Age (year)	64.00 ± 12.10	62.49 ± 9.59	0.676	0.501
Gender (male/female)	15/34	17/32	0.186	0.667
Relevant medical history			4.225	0.238
Diabetes	11 (22.45%)	11 (22.45%)		
Hypertension	24 (48.98%)	19 (38.78%)		
Tumor chemotherapy	12 (24.49%)	11 (22.45%)		

Data was expressed as mean ± SD or *n* (%).

**Table 3:** Comparison of vascular depth and diameter under ultrasound between the two groups.

Group	Blood vessel depth (mm)	Blood vessel diameter (mm)
Control group (*n* = 49)	6.31 ± 0.10	4.65 ± 0.07
Experimental group (*n* = 49)	5.98 ± 0.06	5.23 ± 0.08
*t*	19.81	41.49
*P*	<0.001	<0.001

Data was expressed as mean ± SD.

**Table 4:** Comparison of related indexes of puncture surgery.

Projects	Control group	Experimental group	*t*/*χ*^2^	*P*
One time puncture			9.524	0.002
Successful	36 (73.5%)	47 (95.9%)		
Failed	13 (26.5%)	2 (4.1%)		
Preparation time (min)	2.27 ± 0.19	2.16 ± 0.25	2.452	0.016
Pain response during puncture			7.440	0.004
No pain/slight pain	32 (65.31%)	44 (89.80%)		
Intense pain	17 (34.69%)	5 (10.20%)		
Venipuncture time (min)	18.45 ± 1.26	8.47 ± 1.12	41.110	<0.001
Intravascular congestion postpuncture			5.926	0.015
Yes	20 (40.82%)	9 (18.37%)		
No	29 (59.18%)	40 (81.63%)		
Subcutaneous tissue injury postpuncture			-5.602	<0.001
Needle bleeding	13 (26.53%)	6 (12.24%)		
Subcutaneous bleeding	11 (22.45%)	4 (8.63%)		
Hematoma or stasis	9 (18.37%)	3 (6.12%)		
Vascular reuse rate postpuncture	31 (63.27%)	42 (85.71%)	6.498	0.011
Satisfaction			51.422	≤0.001
Satisfactory	3 (6.12%)	37 (75.51%)		
Generally	34 (69.39%)	12 (24.49%)		
Not satisfactory	12 (24.49%)	0		

Data was expressed as mean ± SD or *n* (%).

## Data Availability

The data used to support the findings of this study are available from the corresponding author upon request.
